This article has been retracted.

# Effect of Intra Uterine Granulocyte Colony Stimulating Factor *vs*. Human Chorionic Gonadotropin at Ovum Pick Up Day on Pregnancy Rate in IVF/ICSI Cases With Recurrent Implantation Failure

**DOI:** 10.5935/1518-0557.20210056

**Published:** 2022

**Authors:** Haitham Torky, El-Sayed El-Desouky, Ashraf El-Baz, Rania Aly, Osama El-Taher, Atef Shata, Ahmed Hussein, Heba Marie, Osama Deif, Ahmed Eldemery, Ashraf Abo-Louz

**Affiliations:** 1 Department of Obstetrics & Gynecology - October 6^th^ University, Giza, Egypt; 2 Department of Obstetrics & Gynecology - Al-Azhar University, Cairo, Egypt; 3 Department of Obstetrics & Gynecology - Al-Galaa Teaching Hospital, Cairo, Egypt; 4 Department of Obstetrics & Gynecology - Matareya Educational Hospital, Cairo, Egypt; 5 Department of Obstetrics & Gynecology - Cairo University, Cairo, Egypt; 6 Department of Biochemistry - October 6^th^ University, Giza, Egypt

**Keywords:** intrauterine injection, G-CSF, hCG, ovum pick-up, clinical pregnancy

## Abstract

**Objective:**

Recurrent implantation failure is defined as failure to achieve clinical pregnancy after the transfer of four or more good-quality embryos in a minimum of three fresh or frozen cycles in a woman aged less than 40 years. The objective is to compare between the effect of intrauterine G-CSF, hCG, and saline solution injection (as placebo) at the day of ovum pick-up on clinical pregnancy, chemical pregnancy, implantation, and miscarriage rates in patients with recurrent implantation failure undergoing IVF/ICSI.

**Methods:**

This prospective, double blind, parallel, randomized controlled trial included 150 patients equally divided into 3 groups, each containing 50 individuals. Subjects in Group 1 received intrauterine injections of G-CSF; Group 2: received intrauterine injections of 500 IU of hCG; and Group 3 received intrauterine injections of saline solution as placebo. The primary outcome measure is clinical pregnancy rate. Secondary outcomes are biochemical pregnancy, implantation, and miscarriage rates.

**Results:**

Clinical pregnancy, biochemical pregnancy, and implantation rates were highest in the group given G-CSF and lowest in the group administered saline solution; miscarriage rates were not significantly different between the groups.

**Conclusions:**

Intrauterine administration of G-CSF at a dose of 100 µg/1.0 cc at the time of ovum pick-up is associated with better clinical pregnancy, chemical pregnancy, and implantation rates as compared with intrauterine saline solution administration. Further studies are needed to determine the optimum timing of intrauterine administration of G-CSF that achieves the best results, and longer follow-up is needed to determine take-home baby percentages.

## INTRODUCTION

Recurrent implantation failure is defined as failure to achieve clinical pregnancy after the transfer of four or more good-quality embryos in a minimum of three fresh or frozen cycles in a woman aged less than 40 years (Coughlan *et al*., 2014). Factors responsible for failure include sperm and oocyte quality, abnormalities in parental chromosomes, metabolic or genetic abnormalities in the embryo, some gynecological conditions (e.g.: hydrosalpinx, endometrial polyps, uterine fibroids), immunological disturbance in the implantation site, and poor endometrial receptivity (Nowak *et al*., 2017).

Several therapies have been described for recurrent implantation failure, including correction of uterine conditions, prescription of antithrombotic agents, and immunotherapy (Bashiri *et al*., 2018). A recently investigated therapy, granulocyte colony-stimulating factor (G-CSF) has been associated with pregnancy success by affecting ovarian function and influencing granulosa cell function to improve ovarian stimulation outcomes in poor responders, enhance embryo implantation, and promote endometrial thickening (Eftekhar *et al*., 2018). Benefits in terms of embryo transfer clinical outcomes are clear when G-CSF is administered systemically or by local infusion (Zhang *et al*., 2018).

Another investigated treatment modality is human chorionic gonadotropin (hCG), an important element in embryo implantation. While intrauterine administration of hCG acts by inhibiting macrophage colony-stimulating factor (M-CSF) and insulin-like growth factor binding protein 1 (IGFBP-1), on the other hand it stimulates vascular endothelial growth factor (VEGF), matrix metalloproteinase (MMP)-9, and leukemia inhibitory factor (LIF), which are important factors in the implantation process (Licht *et al*., 2007). Mansour *et al*. (2011) has further shown that intrauterine injection of 500 IU of hCG before embryo transfer in cases of IVF/ICSI improved both implantation and pregnancy rates.

To our knowledge, this is the first study in which the effects of intrauterine G-CSF, hCG, and saline solution (as placebo) administration at the day of ovum pick-up are compared in terms of clinical pregnancy, chemical pregnancy, implantation and miscarriage rates in patients with recurrent implantation failure undergoing IVF/ICSI.

## MATERIAL AND METHODS

This prospective double blind multicenter parallel randomized controlled trial compared the effects of intrauterine hCG, G-CSF, and saline injection on clinical pregnancy rates as a primary endpoint. The study was conducted in Al-Azhar, October 6^th^ University hospitals, Al-Galaa Teaching Hospital, and private IVF centers between January 2019 and January 2020. The Ethics Committee of Al-Azhar University approved the study, which is in line with the Helsinki Declaration. The study was registered with The Pan-African Clinical Trial Registry and assigned certificate no. PACTR202006915851110.

All patients gave informed consent before joining the trial. The study involved patients aged between 20 and 39 years undergoing IVF/ICSI who had a history of recurrent implantation failure (three or more failed attempts with at least four good quality embryos transferred); women with hypersensitivity or at high risk of developing complications from any of the used medications, with sickle cell nephropathy, with a history of malignancy, with poor quality embryos, and women at risk of ovarian hyperstimulation syndrome (OHSS) were excluded from the study. An independent researcher not involved in the study performed the randomization procedure.

Patients were randomized at the time of ovum pick-up based on a table created using a computer software program with an allocation ratio of 1:1 into three groups, each containing 50 patients. Group 1 included patients given intrauterine injections of G-CSF (Neupogen); Group 2 included patients given intrauterine injections of 500 IU of hCG; and Group 3 included patients given intrauterine injections of saline solution as placebo. Group allocation numbers were delivered in sealed opaque envelopes.

Participants underwent trans-vaginal ultrasound (TVUS) examination on day two of the cycle to assess antral follicle count (AFC), and had FSH, LH, E2, TSH, AMH, and Prolactin levels tested. They were prescribed the long gonadotropin releasing hormone (GnRH) agonist protocol. All patients underwent pituitary desensitization with Decapeptyl 0.1 mg/day (Ferring Pharmaceuticals, Germany) injected subcutaneously from the mid-luteal phase until the day of hCG triggering. After pituitary down-regulation was achieved with serum E2 levels ≤ 50 pg/ml, ovarian stimulation was started from day two of the subsequent menstrual bleeding with daily intramuscular injections of human menopausal gonadotropin (HMG) (Merional 75 IU, IBSA, Switzerland) until the day of hCG injection. Doses of Decapeptyl and HMG were adjusted according to patient age, BMI, and AFC. Ovarian response was monitored through serial transvaginal ultrasound scans performed every three days starting from day six of the cycle. On day six of the cycle, the starting dose of HMG was adjusted according to serum E2 and TVS.

After follicles reached a mean diameter ≥18 mm, the patients were given 10000 IU of highly purified hCG (Choriomon, IBSA Pharmaceutical, Switzerland) - recombinant hCG is not available in the Egyptian market - through intramuscular injection. Oocytes were retrieved 36 hours after hCG injection using a 17-gauge aspiration needle under transvaginal ultrasound guidance.

After oocyte retrieval, G-CSF, 1 cc of Geneleukin 300 µg/1.0 was diluted with dextrose 5% in a ratio of 1:2 and 1 cc containing 100 µg was administrated using the same catheter in subjects in Group 1; hCG for intrauterine injection was prepared diluting one vial containing 5,000 IU of hCG (Choriomon, IBSA Pharmaceutical, Switzerland) in 10 cc of normal saline solution, so that each 1 cc contained 500 IU of hCG, which was later injected using a Wallace embryo replacement soft catheter (Smiths Medical International Ltd., UK) in subjects in Group 2; 1 cc of normal saline solution was injected in subjects in Group 3. The catheter was left *in situ* for 15 minutes to ensure that there was no leakage of the injected fluid. The pelvis was evaluated with ultrasound to make sure there was no internal bleeding. All the medications in all groups were prepared by the attending specialist registrar and handled to the participating physician who was blinded to the injected medication. All patients were asked to remain in the lithotomy position for half an hour before being discharged.

After fertilization, one to three grade-A embryos (maximum number allowed in Egypt), rated as optimum quality embryos with the best chance of implantation according to ASEBIR criteria for embryo grading (ASEBIR, 2015), were transferred on day five fertilization. Luteal phase support was initiated on the day of oocyte retrieval for all patients with daily Cyclogest 400 mg (Actavis pharmaceutical, UK) vaginal suppositories until the day the patients underwent serological testing for pregnancy. Serum β-hCG was measured 14 days after embryo transfer, and clinical pregnancy was confirmed when there was evidence of gestational sac, embryo, and fetal heart activity at time of transvaginal ultrasound examination by the 8^th^ week.

The primary endpoint of the study was clinical pregnancy rate (defined as viable pregnancy with evidence of gestational sac, embryo, and fetal heart activity at the time of transvaginal ultrasound evaluation by the eighth week); secondary endpoints included biochemical pregnancy rate (defined as positive from quantitative values of serum β-hCG levels according to the standard values used in the laboratory), implantation rate (defined as the number of gestational sacs observed during ultrasound screening at 6 weeks of pregnancy divided by the number of embryos transferred), and miscarriage rate (defined as the loss of pregnancy before the 8^th^ week of gestation).

### Statistical analysis

Recorded data were analyzed using the Statistical Package for Social Sciences, version 20.0 (SPSS Inc., Chicago, Illinois, USA). Quantitative data were expressed as mean ± standard deviation (SD). Qualitative data were expressed as frequencies and proportions.

The following tests were performed:

• One-way analysis of variance (ANOVA): comparisons between more than two means.
• Post Hoc test: Least Significant Difference (LSD) was used for multiple comparisons between different variables.
• Kruskal-Wallis test: multiple-group comparisons of non-parametric data.
• Chi-squared (x^2)^ test of significance: comparisons between proportions and qualitative parameters.
• The confidence interval was set at 95% and the margin of error accepted was set at 5%. Therefore, the p-value was considered significant as follows:
• Probability (*p*-value):
- *p*-value <0.05 was considered significant.
- *p*-value <0.001 was considered highly significant.
- *p*-value >0.05 was considered insignificant.

### Sample size calculation

MedCalc^®^ version 12.3.0.0 (Ostend, Belgium) was used in sample size calculations, statistical calculator based on 95% confidence interval, and power of the study at 80% with α error 5%*.* A previous study (Mostafa & Farid, 2017) reported clinical pregnancies in 22% of the patients given G-CSF and in 16% of the women in the control group, with a significant difference between the two groups (*p*-value <0.05). Based on the findings published in this study, the minimum sample size calculated to find such difference was 95. Assuming a dropout ratio of 5%, the sample size should be 50 women in each of the two groups. We added another group and the number went up to 150, subdivided into three groups; G-CSF (n=50), hCG (n=50), and Saline Solution (n=50).

## RESULTS

Table 1 shows the basic demographic information of study participants.

**Table 1.** Comparison between groups according to demographic data.

Demographic data	G-CSF (n=50)	hCG (n=49)	Saline (n=48)	Test	*p*-value
**Age (years)** Mean±SD Median (Range)	35.1±5.04 36 (23-43)	35.33±5.11 37 (24-44)	35.17±4.23 36 (25-43)	H=0.245	0.885
**Weight (kg)** Mean±SD Median (Range)	87.12±17.42 90 (54-111)	85.67±17.03 88 (52-122)	84.25±9.45 87 (54-96)	H=2.390	0.303
**Height (m)** Mean±SD Median (Range)	1.71±0.08 1.7 (1.62-1.87)	1.71±0.08 1.7 (1.5-1.85)	1.71±0.0 1.7 (1.62-1.85)	H=0.161	0.923
**Husband Age (years)** Mean±SD Median (Range)	40.38±7.11 40 (30-59)	40.96±7.07 40 (27-53)	38.94±3.9 39 (31-50)	H=2.416	0.299
**Duration of Infertility (years)** Mean±SD Range	6.27±2.49 5.5 (3-12)	6.63±2.74 6 (4-13)	6.69±2.72 7 (3-12)	H=0.656	0.720
**Type of Infertility** Primary Secondary	38 (76.0%) 12 (24.0%)	38 (77.6%) 11 (22.4%)	31 (64.6%) 17 (35.4%)	x2=2.453	0.293
**Cause of infertility** Male Ovarian Polycystic ovary Tubal Unexplained	9 (18.0%) 2 (4.0%) 9 (18.0%) 7 (14.0%) 23 (46.0%)	15 (30.6%) 4 (8.2%) 3 (6.1%) 8 (16.3%) 19 (38.8%)	14 (29.2%) 2 (4.2%) 8 (16.7%) 8 (16.7%) 16 (33.3%)	x^2^=7.022	0.534
**Previous IVF/ICSI** Mean±SD Median (Range)	3.7±1.09 3 (3-6)	4.43±0.94 4 (4-7)	3.67±0.81 3 (3-5)	H=26.147	<0.001*

H- Kruskal-Wallis Test; x^2^: Chi-squared test; *p*-value >0.05 NS;

* *p*-value <0.05 is significant.

Table 2 compares the baseline hormonal profiles (FSH, LH, E2, AMH, Prolactin and TSH), antral follicle counts, baseline endometrial thicknesses, and endometrial thicknesses at the time of embryo transfer see in each group.

**Table 2.** Comparison between groups according to baseline hormonal profile (FSH, LH, E2, AMH, Prolactin and TSH), antral follicle count, baseline endometrial thickness, and endometrial thickness at embryo transfer.

Variables	G-CSF (n=50)	hCG (n=49)	Saline (n=48)	Test	*p*-value
**FSH mIU/ml** Mean±SD Median (Range)	6.46±1.73 6.5 (2.5-10)	6.92±1.31 6.5 (5.5-10)	7.24±1.7 7.2 (4.9-10)	H=1.717	0.424
**LH mIU/ml** Mean±SD Median (Range)	0.9±0.55 0.9 (0.1-2.8)	0.78±0.67 0.5 (0.1-2.8)	0.9±0.72 0.8 (0.1-2.8)	H=3.377	0.185
**E2 pgm/ml** Mean±SD Median (Range)	38.56±12.24 38.5 (18-60)	37.92±13.06 42 (5-52)	34.85±13.6 31 (18-56)	H=2.187	0.335
**AMH ng/ml** Mean±SD Median (Range)	2.08±1.08 1.9 (0.8-4.2)	2±1.12 1.8 (0.1-4.9)	1.96±0.83 1.9 (0.9-4.1)	H=0.026	0.987
**Prolactin mIU/ml** Mean±SD Median (Range)	23.26±7.47 24 (10-32)	21.94±6.87 22 (7-31)	24.71±5.89 26.5 (17-32)	H=4.175	0.124
**TSH uIU/l.** **Mean**±SD Median (Range)	2.68±0.93 2.85 (0.1-4.9)	2.58±0.86 2.7 (0.6-4.8)	2.65±1.18 2.75 (0.1-4.9)	H=0.304	0.859
**Antral follicle count** Mean±SD Median (Range)	9.2±3.62 8 (4-14)	9.55±3.15 9 (4-17)	9.5±2.49 10 (5-14)	H=0.979	0.613
**Endometrial Thickness baseline** Mean±SD Median (Range)	4.88±5.28 4.3 (2.8-41.1)	5.38±6.23 4.2 (2.5-35)	5.59±7.51 4 (2.9-41.1)	H=0.649	0.723
**Endometrial Thickness at embryo transfer** Mean±SD Median (Range)	9.87±1.61 9.35 (7.3-13)	9.89±2.2 9.4 (2.7-16)	10.31±1.53 10 (8-13)	H=2.811	0.245

H- Kruskal-Wallis Test; *p*-value >0.05 NS

Table 3 describes cycle day of hCG trigger, timing of oocyte retrieval, and gonadotropin doses in all groups.

**Table 3.** Comparison between groups according to cycle day of hCG trigger dose, timing of oocyte retrieval, and gonadotropin dose

Variables	G-CSF (n=50	hCG (n=49)	Saline (n=48)	Test	*p*-value
**hCG trigger dose (day of cycle)** D9 D10 D11 D12 D13	7 (14.0%) 20 (40.0%) 8 (16.0%) 8 (16.0%) 7 (14.0%)	3 (6.1%) 22 (44.9%) 9 (18.4%) 9 (18.4%) 6 (12.2%)	5 (10.4%) 21 (43.8%) 9 (18.8%) 8 (16.7%) 5 (10.4%)	x^2^=2.127	0.977
**Oocyte Retrieval (Hours after hCG trigger)** 33 Hours 34 Hours 35 Hours 36 Hours 37 Hours 38 Hours 39 Hours	1 (2.0%) 1 (2.0%) 4 (8.0%) 39 (78.0%) 3 (6.0%) 0 (0.0%) 2 (4.0%)	0 (0.0%) 2 (4.1%) 7 (14.3%) 37 (75.5%) 2 (4.1%) 1 (2.0%) 0 (0.0%)	0 (0.0%) 1 (2.1%) 6 (12.5%) 37 (77.1%) 3 (6.3%) 1 (2.1%) 0 (0.0%)	x^2^=8.524	0.743
**Gonadotropin Dose, IU** Mean±SD Median (Range)	35.28±6.17 33 (28-50)	35.86±5.29 36 (27-45)	37.33±6.14 37 (30-50)	H=3.452	0.178

x^2^: Chi-squared test; H- Kruskal-Wallis Test; *p*-value >0.05 NS

Table 4 compares the number of retrieved oocytes, metaphase II oocytes, and embryos transferred in each group.

**Table 4.** Comparison between groups according to number of retrieved oocytes, number of metaphase II oocytes, and number of transferred embryos.

Variables	G-CSF (n=50)	hCG (n=49)	Saline (n=48)	Test	*p*-value
**Retrieved oocytes** Mean±SD Median (Range)	10.8±4.94 10 (3-24)	10.24±5.74 8 (1-22)	9.92±4.13 9.5 (3-24)	H=1.116	0.572
**Metaphase II oocytes** Mean±SD Median (Range)	7.1±4 6.5 (1-18)	6.92±4.83 5 (1-18)	6.75±3.7 7 (1-18)	H=0.318	0.853
**No. of transferred embryos** Mean±SD Median (Range)	2.46±0.71 3 (1-3)	2.39±0.81 3 (1-3)	2.35±0.67 2 (1-3)	H=0.899	0.638

H- Kruskal-Wallis Test; *p*-value >0.05 NS

Table 5 compares between the different study outcomes (clinical and chemical pregnancy rates; implantation and miscarriage rates) seen in the groups.

**Table 5.** Comparison between groups according to endpoints chemical pregnancy, clinical pregnancy, implantation, and miscarriage rates.

Variables	G-CSF (n=50)	hCG (n=49)	Saline (n=48)	Test	*p*-value
**Chemical Pregnancy**	29 (58%)	24 (49%)	13 (27.1%)	x2=9.738	0.007*
**Clinical Pregnancy**	28 (56%)	23 (46.9%)	11 (22.9%)	x2=11.863	0.003*
**Implantation rate**	43/123 (35%)	28/120 (23.3%)	16/118 (13.6%)	x2=15.136	<0.001*
**Miscarriage**	1 (2%)	1 (2.04%)	2 (4.2%)	x2=0.563	0.755

x^2^: Chi-squared test;

* *p*-value <0.05 is significant;

*p*-value >0.05 NS.

One patient in Group 2 and two in Group 3 were lost during follow-up.

There were 11 twin pregnancies and two triplet pregnancies in the G-CSF group; one twin pregnancy and one triplet pregnancy was recorded in Group 2; three twin pregnancies and one triplet pregnancy were seen in the group given saline solution.

There were no cases of ectopic pregnancy.

## DISCUSSION

The present study showed that intrauterine administration of G-CSF or hCG at the time of oocyte retrieval yielded significantly higher clinical pregnancy, chemical pregnancy, and implantation rates as compared with intrauterine saline solution (placebo) in women with recurrent implantation failure; G-CSF administration produced better results than hCG in regard to the same outcomes; miscarriage rates did not differ significantly between the three groups. The lower implantation (13.9%) and pregnancy rates (chemical pregnancy rate of 27.1% and clinical pregnancy rate of 22.9%) seen in the saline solution group may be explained by the negative effect of saline solution injection in patients with recurrent implantation failure, as previously published (Salehpour *et al*., 2016) in a study in which the effect of intrauterine saline infusion in fresh IVF cycles was analyzed as a form of endometrial injury. The authors found that saline solution produced negative effects on reproductive outcomes (lower pregnancy and implantation rates) in women with recurrent implantation failure.

The results of the present study agreed with the results of several other studies (Mansour *et al*., 2011; Gao *et al*., 2019; Navali *et al*., 2016). The first study by Mansour *et al*. (2011) looked into the intrauterine administration of 500 IU of hCG at the time of embryo transfer in women aged less than 40 years and found higher clinical pregnancy and implantation rates as compared to not administering hCG to women undergoing IVF/ICSI for the first time. The second study by Gao *et al*. (2019) was a meta-analysis of 15 randomized controlled trials including 2763 patients. The authors concluded that intrauterine injection of hCG improved live birth, ongoing pregnancy, clinical pregnancy, and implantation rates in patients undergoing IVF cycles. The third study by Navali *et al*. (2016) was a randomized controlled trial - similar in timing, dose and route of hCG administration to the present study - that included 158 patients on the antagonist protocol, who received either intrauterine administration of 500 IU hCG or normal saline solution right after oocyte retrieval. The authors found that intrauterine administration of hCG immediately after oocyte retrieval increased the implantation, chemical, and clinical pregnancy rates of individuals given intrauterine hCG.

The results of the present study also agreed with the results published by Tapilskaya *et al*. (2019), which discussed four different meta-analyses exploring the efficacy of administering G-CSF to infertile women undergoing IVF. The authors found increases in implantation and clinical pregnancy rates attributed to changes in endometrial receptivity and/or invasive potential of the developing embryo. However, our results differed from the ones reported by Zafardoust *et al*. (2017) in a randomized controlled trial designed to study the effects of G-CSF in women with recurrent miscarriage (at least two) on clinical pregnancy and miscarriage rates. The authors did not find a significant difference in either of the parameters. This discrepancy may be attributed to the dose used in their study, which was 300 microgram of G-CSF, i.e., three times the dose used in the present study, showing a possible dose-dependent response for G-CSF. Cavalcante *et al*. (2020) pointed to the latter in a systematic review devised to evaluate intrauterine perfusion immunotherapies in patients with recurrent implantation failure. The authors concluded that the results were encouraging despite the limited number of studies published on the subject. However, there is still a lack of uniform protocols and doses for this kind of therapy due to discrepancies in the protocols used in these studies.

The present study found significantly greater numbers of multiple pregnancies, namely twin pregnancies, in the G-CSF group as compared with the other two groups. The difference may be attributed to the significantly higher implantation rates in the G-CSF group. However, only a few of the studies on the subject reported multiple pregnancy rates. Kalem *et al*. (2020) described five twin pregnancies in individuals given G-CSF compared to controls, although the dose of G-CSF used in their trial was much lower than the one used in our study (30 mIU/mL of Leucostim).

In regards to the safety of G-CSF on the developing embryo, several studies have looked into the effects of G-CSF in pregnant patients with cancer and found no significant difference in teratogenicity between patients prescribed G-CSF and individuals not prescribed G-CSF, thereby indicating that G-CSF had no teratogenic effect on the developing fetus (Zeidler *et al*., 2014; Boxer *et al*., 2015; Gurevich-Shapiro & Avivi, 2019; Cardonick *et al*., 2012).

The advantages of the present study include adequate study power and the fact that this has been the first study, to our knowledge, to directly compare the effect of intrauterine G-CSF and hCG administration on clinical pregnancy, biochemical pregnancy, implantation, and miscarriage rates. The limitations of the study include the determination of the best time to administer G-CSF to reach its maximum effect, and the long term follow-up of the women who got pregnant to calculate take-home baby rates.

## CONCLUSION

Intrauterine administration of G-CSF at a dose of 100 µg/1.0 cc at the time of ovum pick-up is associated with better clinical pregnancy, chemical pregnancy, and implantation rates than intrauterine saline solution administration. Further studies are needed to determine the optimum timing of intrauterine administration of G-CSF to achieve the best results; longer follow-up is needed to determine take-home baby rates.
